The article "The causal relationships of granulocytes and melanoma skin cancer: A univariable and multivariable Mendelian randomization study" was retracted in 2025. Reasons: unreliable results or conclusions; concerns about the methods; concerns about the peer review.

# The causal relationships of granulocytes and melanoma skin cancer: A univariable and multivariable Mendelian randomization study

**DOI:** 10.1111/srt.70007

**Published:** 2024-08-16

**Authors:** Zhang Rui‐chang, Peng Hui‐zi, Zhou Lin

**Affiliations:** ^1^ Department of Cosmetic Maxillofacial Surgery the First Affiliated Hospital of Xi'an Jiaotong University Xi'an Shannxi China

**Keywords:** causal relationship, eosinophil percentage, GWAS, melanoma skin cancer, mendelian randomization neutrophil percentage

## Abstract

**Background:**

Increasing evidence has revealed that granulocyte has a critical role in tumorigenesis and progression. In this study, Mendelian randomization (MR) analysis was utilized for estimating the causal association between neutrophil percentage and melanoma skin cancer, eosinophil percentage and melanoma skin cancer, basophil percentage and melanoma skin cancer, respectively.

**Methods:**

The Genome‐Wide Association Study (GWAS) ids for melanoma skin cancer, neutrophil percentage, eosinophil percentage and basophil percentage were derived from Integrative Epidemiology Unit (IEU) Open GWAS database. The univariable MR (UVMR) analysis was conducted to estimate the risk using MR‐Egger, weighted median, inverse variance weighted (IVW). In addition, sensitivity analysis was conducted to assess the reliability of UVMR results. Finally, the multivariable MR (MVMR) analysis was performed to investigate causality between neutrophil percentage and eosinophil percentage in the presence of both and melanoma skin cancer.

**Results:**

The UVMR indicated that neutrophil percentage and eosinophil percentage were significantly and causally related to melanoma skin cancer, with neutrophil percentage [*p* = 0.025, odds ratio (OR) = 1.002] as a risk factor and eosinophil percentage (*p* = 7.04E‐06, OR = 0.997) as a protective factor. Moreover, MVMR analysis indicated eosinophil percentage remained the protective factor (*p* = 0.003, OR = 0.998), while the causality of neutrophil percentage and melanoma skin cancer became insignificant (*p* > 0.05).

**Conclusion:**

The causal relationships of neutrophil percentage and melanoma skin cancer, eosinophil percentage and melanoma skin cancer were shown by this study, which provided a reference for subsequent research and treatment related to melanoma skin cancer.

## 1 INTRODUCTION

Melanoma skin cancer (cutaneous melanoma) represents a highly aggressive and potentially fatal form of cancer stemming from melanocytes.^1^ Insights from molecular biology and advanced sequencing techniques have underscored the predominant role of genetic and environmental factors in melanoma skin cancer etiology. Despite constituting only 4% of skin cancer diagnoses, melanoma skin cancer is responsible for a staggering 75% of skin cancer‐related deaths.^2^, ^3^ According to the GLOBOCAN 2020 database, there were 324 635 new cases of melanoma and 57 043 deaths in 185 countries worldwide in 2020.^4^ Recent studies suggest that timely detection and appropriate intervention can significantly reduce the mortality rate of melanoma skin cancer. Therefore, the timely detection and prognosis of melanoma emerge as pivotal areas warranting heightened attention and focus.

The article "The causal relationships of granulocytes and melanoma skin cancer: A univariable and multivariable Mendelian randomization study" was retracted in 2025. Reasons: unreliable results or conclusions; concerns about the methods; concerns about the peer review.

Numerous potential biomarkers have been utilized to evaluate the prognosis and therapeutic effect of melanoma.^5^ However, many of these tests are cumbersome, costly, and yield inconsistent results, which has limited their use in clinical practice. The granulocyte in peripheral smear test, due to its ease and affordability, has been studied for its potential prognostic value in melanoma assessment.^6^, ^7^, ^8^ Neutrophils, as the most abundant immune cells in the tumor microenvironment, release specific pro‐tumoral factors.^9^, ^10^ Eosinophils are recruited in the peripheral blood of tumor patients, and their levels correlate with patient survival.^11^ Basophils account for a smaller proportion of the population but can recruit CD8^+^ T cells to infiltrate, exhibiting potential anti‐tumor properties. Previous research has shown that the neutrophil/lymphocyte ratio (NLR) is linked to improved overall survival rates among melanoma patients receiving immune checkpoint inhibitors.^12^ In addition, Pozorski^13^ demonstrated that the neutrophil/eosinophil ratio (NER) can be used as a new prognostic marker in advanced melanoma patients receiving anti‐PD‐1 therapy. Further investigation is therefore needed into the relationship between granulocyte and melanoma prognosis.

Mendelian randomization (MR) estimates causal effects of exposure and outcome using germline genetic variation as an instrumental variable. Because alleles assort randomly during meiosis and germline genetic variation is fixed at conception, the analysis is immune to conventional confounding and reverse causality in epidemiological observations.^14^ Genetic evidence for the effect of exposure changes (e.g., granulocyte percentage) on outcome (e.g., melanoma skin cancer prognosis) can therefore be provided by MR studies. To date, no comprehensive MR study of the association between peripheral blood neutrophils/eosinophils/basophils and melanoma prognosis has been reported.

In this study, a univariate and multivariate MR study was performed based on genetic variation data from public databases for melanoma skin cancer and the three exposure factors (eosinophil percentage, neutrophil percentage, and basophil percentage) to investigate the causal effect of granulocyte on melanoma skin cancer, and sensitivity analyses were performed to assess the impact of assumptions on findings and to ensure the robustness of results.

The article "The causal relationships of granulocytes and melanoma skin cancer: A univariable and multivariable Mendelian randomization study" was retracted in 2025. Reasons: unreliable results or conclusions; concerns about the methods; concerns about the peer review.

## 2 MATERIALS AND METHODS

### 2.1 Data source

The Genome‐Wide Association Study (GWAS) ids for melanoma skin cancer (ieu‐b‐4969), neutrophil percentage (id:ukb‐d‐30200_irnt), eosinophil percentage (id:ukb‐d‐30210_irnt), and basophil percentage (id:ukb‐d‐30220_irnt) were derived from Integrative Epidemiology Unit (IEU) Open Genome‐Wide Association Study (GWAS) database (https://gwas.mrcieu.ac.uk/). The ieu‐b‐4969 dataset (3751 melanoma skin cancer samples and 372 016 control samples) contained 11 396 019 single nucleotide polymorphisms (SNPs). The sample size for ukb‐d‐30200_irnt dataset was 349 861, and the number of SNPs was 13 586 283. In this study, neutrophil percentage, eosinophil percentage, and basophil percentage were the exposure factors, and melanoma skin cancer was the outcome variable.

### 2.2 Selection of instrumental variables (IVs)

Three fundamental premises served as the foundation for the MR study: (1) there was a significant correlation between IVs and exposure; (2) the IVs were independent of confounders; (3) the IVs could only influence the outcome through exposure and not through any other channels.

In this study, SNPs (IVs) were selected (*p* < 5*10^−8^) using “TwoSampleMR” R package (version 0.5.6).^15^ Independent SNPs closely associated with neutrophil percentage, eosinophil percentage, and basophil percentage were scanned. IVs were clumped for linkage disequilibrium analysis (LDA) to ensure independence (*r* ^2^ = 0.001 and kb = 10 000).

### 2.3 Univariable MR (UVMR) and sensitivity analysis

The input data for UVMR analysis was taken after filtering the IVs. The major MR modes were MR‐Egger,^16^ simple mode, weighted mode,^17^ weighted median,^18^ and inverse variance weighted (IVW) regression.^19^ The most important method was IVW in this study. Odds ratio (OR) was then calculated, with greater than 1 representing a risk factor and less than 1 representing a protective factor. The results were presented using scatter plots, forest plots, and funnel plots.

Sensitivity analyses were conducted to assess the reliability of UVMR results, which mainly consisted of the heterogeneity test, horizontal pleiotropy test and leave‐one‐out (LOO) analysis. First, Cochran's Q‐test was conducted, and there was no heterogeneity when the *p‐*value was greater than 0.05. Second, potential horizontal pleiotropy among IVs was evaluated using MR‐Egger test, and when *p* was greater than 0.05, it indicated no horizontal pleiotropy, meaning that there was no confounding factors in the study. Finally, LOO analysis was conducted to check whether the UVMR results were influenced by any single SNP.

The article "The causal relationships of granulocytes and melanoma skin cancer: A univariable and multivariable Mendelian randomization study" was retracted in 2025. Reasons: unreliable results or conclusions; concerns about the methods; concerns about the peer review.

### 2.4 Multivariable MR (MVMR) analysis

To examine the causal relationship between neutrophil percentage and melanin skin cancer, between eosinophil percentage and melanin skin cancer, respectively, at a multivariate level, MVMR analysis was applied. The data processing for MVMR analysis was equivalent to UVMR (*p* < 5*10^−8^, *r* ^2^ = 0.001, kb = 10 000).

## 3 RESULTS

### 3.1 Connection of neutrophil percentage, eosinophil percentage, and basophil percentage to melanoma skin cancer

After screening, 262 SNPs for neutrophil percentage, 296 SNPs for eosinophil percentage and 101 SNPs for basophil percentage independent SNPs were obtained as IVs. Table S1 listed the MR results of five different methods. The IVW results showed that neutrophil percentage (*p* = 0.025) and eosinophil percentage (*p* = 7.04E‐06) were causally associated with melanoma skin cancer. However, melanoma skin cancer was not directly related to basophil percentage (*p* = 0.706). Observation of OR values revealed that neutrophil percentage (OR = 1.002) was a risk factor and eosinophil percentage (OR = 0.997) was a protective factor for melanoma skin cancer (Figure 1). The scatter plots showed that slope of the line for neutrophil percentage was positive, indicating that increased amount of neutrophil percentage led to increased risk of melanoma skin cancer, and slope of the line for eosinophil percentage showed an opposite trend to neutrophil percentage, indicating that eosinophil percentage was a protective factor for melanoma skin cancer (Figure 2). The SNPs locations in the forest plots were protection on the left and risk on the right. Our findings supported that neutrophil percentage was a risk factor and eosinophil percentage was a protective factor for melanoma skin cancer (Figures S1 and S2). Also, the funnel plots demonstrated that UVMR analysis conformed to Mendel's second law of random grouping (Figure S3).

**FIGURE 1:** Forest plot showing the MR results of five different methods between melanoma skin cancer risk and neutrophil (A), eosinophil (B), basophil percentage (C). The IVW results showed that neutrophil percentage (*p* = 0.025) and eosinophil percentage (*p* = 7.04E‐06) were causally associated with melanoma skin cancer. The OR values for all five methods were in the same direction and all greater than 1, indicating that the percentage of neutrophils is a risk factor for melanoma skin cancer. Conversely, eosinophils have a protective effect.

The article "The causal relationships of granulocytes and melanoma skin cancer: A univariable and multivariable Mendelian randomization study" was retracted in 2025. Reasons: unreliable results or conclusions; concerns about the methods; concerns about the peer review.

**FIGURE 2:** MR‐Egger scatter plot of melanoma skin cancer risk with neutrophil percentage (A) and eosinophil percentage (B).

### 3.2 UVMR analysis results were proven to be reliable through sensitivity analyses

Sensitivity analyses were carried out to determine the reliability of analysis. The *p‐*values of Cochran's Q‐test were all less than 0.05, indicating that there was heterogeneity among the selected SNPs (Tables 1 and 2). Although there was heterogeneity, the *p‐*value of the IVW method were all less than 0.05, indicating that the heterogeneity did not significantly affect the results of UVMR analysis, which meant that the results of UVMR analysis were valid. The results of MR‐Egger test suggested that there were no horizontal pleiotropy effect among IVs (*p* > 0.05) in UVMR analysis (Table 3). Meanwhile, the intercept values were all less than 0.01, which meant that there were no confounding factors in our analysis. Furthermore, there was no point of serious bias in the results of LOO analyses, indicating that the UVMR analysis results were reliable (Figures S4 and S5). In conclusion, neutrophil percentage and eosinophil percentage were causally associated with development of melanoma skin cancer, with neutrophil percentage as a risk factor and eosinophil percentage as a protective factor for melanoma skin cancer.

**TABLE 1:** The heterogeneity of neutrophil instrumental variables.

Exposure	Outcome	Method	Q	df	*p*
Neutrophil percentage	Melanoma skin cancer	MR Egger	323.650	260	0.004*
Neutrophil percentage	Melanoma skin cancer	Inverse variance weighted	323.651	261	0.005*

*Note*:*p<*0.05*, indicating that the heterogeneity between the neutrophil percentage and melanoma skin cancer datasets did not significantly affect the analysis results, which meant the analyses were valid.

**TABLE 2:** The heterogeneity of eosinophil instrumental variables.

Outcome	Exposure	method	Q	df	*p*
Melanoma skin cancer	Eosinophil percentage	MR Egger	376.717427	294	0.000782844*
Melanoma skin cancer	Eosinophil percentage	Inverse variance weighted	377.0937669	295	0.00085678*

*Note*:*p<*0.05*, indicating that the heterogeneity between the eosinophil percentage and melanoma skin cancer datasets did not significantly affect the analysis results, which meant the analyses were valid.

**TABLE 3:** Horizontal pleiotropy assessed of the association between neutrophil/eosinophil and melanoma skin cancer.

Outcome	Exposure	Egger_intercept	SE	*p*
Melanoma skin cancer	Neutrophil percentage	1.30E‐06	4.38E‐05	0.976419
Melanoma skin cancer	Eosinophil percentage	−2.02E‐05	3.73E‐05	0.588266

### 3.3 Relationship between neutrophil percentage and eosinophil percentage in the presence of both and melanoma skin cancer by MVMR analysis

After screening, 302 SNPs associated with neutrophil percentage and eosinophil were identified and taken as input data for MVMR analysis. No changes in the protective or risk properties of two exposure factors were observed after the assessments (Figure 3, Table S2). However, the *p*‐value for neutrophil percentage was greater than 0.05, meaning the causality between neutrophil percentage and melanoma skin cancer became insignificant. In other words, the influence of eosinophil percentage as a protective factor for melanoma skin cancer was more direct than neutrophil percentage.

The article "The causal relationships of granulocytes and melanoma skin cancer: A univariable and multivariable Mendelian randomization study" was retracted in 2025. Reasons: unreliable results or conclusions; concerns about the methods; concerns about the peer review.

**FIGURE 3:** Forest plot for MVMR analysis of melanoma skin cancer with neutrophil percentage and eosinophil percentage. The *p*‐value for eosinophil percentage remained below 0.05, indicating a more direct impact on melanoma skin cancer.

## 4 DISCUSSION

Melanoma skin cancer stands as the most lethal form of cutaneous malignancy.^20^ It is imperative to establish a straightforward and efficient method for early diagnosis and prognosis assessment of melanoma.^21^ Immune checkpoint inhibitor (ICI)‐based therapies (especially those targeting anti‐cytotoxic T‐lymphocyte‐associated antigen‐4 (anti‐ctla‐4) and anti‐programmed death‐1 (anti‐pd‐1) antibodies) have dramatically improved overall survival in melanoma in recent years,^22^ but unfortunately, there are still no validated biomarkers to indicate the therapeutic prognosis of ICL. Given the simplicity and convenience of peripheral blood tests, coupled with the pivotal role of granulocytes in tumorigenesis and progression, we aimed to investigate the significance of peripheral blood granulocyte percentage in the prognostic determination of melanoma.^23^

Studying correlations can be challenging due to the complex and time‐consuming design of prospective studies. Additionally, changes in granulocytes in peripheral blood are associated with various factors, which can lead to biased epidemiological studies. Therefore, providing strong evidence can be difficult. It is important to acknowledge the limitations of traditional epidemiological studies. Due to the potential for bias in experimental designs and clinical studies, the causal relationship between exposure and disease can often be influenced by confounding factors. To address this issue, MR analysis offers a new approach for assessing the causal relationship between exposure and disease by using genetic variation.^24^ Genetic variants can be used as a randomized controlled trial (RCT) because they are assigned to individuals before any exposure or outcome occurs, and this assignment is randomized. This reduces the occurrence of reverse causation and potential confounders, making the results similar to those of an RCT.^24^, ^25^

Previous studies have employed MR to investigate the crucial role of inflammation‐related factors in the progression of certain skin diseases and malignant tumors.^26^, ^27^ This study presents the first MR analysis to investigate the causal relationship between the percentage of neutrophils and eosinophils in peripheral blood and prognosis in melanoma. It is the largest and most comprehensive study of its kind to date.

The article "The causal relationships of granulocytes and melanoma skin cancer: A univariable and multivariable Mendelian randomization study" was retracted in 2025. Reasons: unreliable results or conclusions; concerns about the methods; concerns about the peer review.

Our study found a significant causal effect of neutrophil percentage on melanoma skin cancer and that neutrophil percentage was a risk factor. It is well known that lymphocytes have a well‐established anti‐tumor role, and their immune surveillance and destruction of neoplastic tumors are essential. With respect to neutrophils, it can inhibit lymphocyte proliferation and induce lymphocyte apoptosis. It is widely accepted that neutrophils are positively correlated with tumor progression,^9^, ^28^, ^29^ which is consistent with our findings. Neutrophils expressing PD‐L1 can induce T‐cell apoptosis by binding to lymphocyte PD‐1.^30^ In addition, neutrophils can directly reduce lymphocyte proliferation by producing reactive oxygen species and arginase‐1. Furthermore, neutrophil extracellular traps (NETs) have been shown to enhance tumor cell adhesion and promote extracellular matrix degradation, thereby facilitating tumor metastasis.^31^, ^32^ Based on this, numerous studies have investigated the reliability of the neutrophil‐to‐lymphocyte ratio (NLR) as a means of determining the prognosis of melanoma.^33^ A meta‐analysis of 12 studies and 3207 patients^34^ with stage I‐IV melanoma revealed that a high NLR is independently associated with higher melanoma‐specific mortality, leading to significantly worse overall survival. However, Wade et al.^35^ conducted a multicenter cohort study with a total of 1351 patients (66% stage I) and found that high NLR was positively associated with better overall survival and disease‐free survival. In the early stages of melanoma, neutrophils have been found to be more anti‐tumor. Further studies have confirmed that the main regulator of the pro‐ or anti‐tumorigenic neutrophil phenotype is Notch1, which is elevated to a greater extent in advanced melanoma.^36^

Furthermore, there was a significant causal relationship between eosinophil percentage and melanoma skin cancer in our study, and eosinophil percentage was a protective factor for the risk of melanoma skin cancer.^37^, ^38^ Research on the relationship between eosinophils and melanoma prognosis is limited. However, existing studies indicate that eosinophils have anti‐tumor effects for most types of cancer, including melanoma, again in agreement with our findings. Research has shown that eosinophils produce chemokines, including CCL5, CXCL9, and CXCL10, which attract reactive CD8+ T cells to the tumor microenvironment^11^. Additionally, eosinophils have the ability to directly kill tumor cells. Ferrucci et al. found that baseline relative eosinophil counts can serve as a predictive biomarker for the anti‐PD‐1 treatment of advanced melanoma.^39^, ^40^

What is more, after conducting a MVMR analysis, it was found that the *p*‐value of neutrophil percentage was greater than 0.05, indicating that the causal relationship between neutrophil percentage and melanoma skin cancer became insignificant. Therefore, the effect of eosinophil percentage as a protective factor for melanoma skin cancer is more direct than that of neutrophil percentage. This partially supports prior research indicating that neutrophils play distinct roles during various stages of melanoma development. They may exhibit anti‐tumor properties during the early stages of tumor growth, but overall, they still exhibit tumorigenic properties. In contrast, eosinophils demonstrate more direct anti‐tumor properties, and a higher percentage of eosinophils suggests a better prognosis for melanoma.

The article "The causal relationships of granulocytes and melanoma skin cancer: A univariable and multivariable Mendelian randomization study" was retracted in 2025. Reasons: unreliable results or conclusions; concerns about the methods; concerns about the peer review.

There are limitations to this study. Firstly, the data analyzed were mainly from populations of European origin. Therefore, a larger sample of multiethnic groups with more relevant SNPs may have contributed to more reliable conclusions. Secondly, due to the limitations of the sample and clinical data, subgroup analyses were not possible. For example, the role of neutrophils at different stages of tumor development remains unclear. This prevented us from using MR to gain further insight into the study for clinical purposes.

## 5 CONCLUSION

Our study have shown a potential causal relationship between the percentage of eosinophils and neutrophils with melanoma skin cancer using UVMR. However, the MVMR analysis did not find a significant causal relationship between neutrophil percentage and melanoma skin cancer. On the other hand, eosinophil percentage remained a direct protective factor against melanoma. The data suggests that a decrease in eosinophil percentage is directly associated with the development of melanoma skin cancer, while altered neutrophil percentage may not be directly associated with it. Therefore, it is important to monitor the eosinophil percentage of patients and consider it in the prognosis of melanoma skin cancer. Early targeted treatment should be considered based on this information.

## CONFLICT OF INTEREST STATEMENT

The authors declare that they have no competing interests.

The article "The causal relationships of granulocytes and melanoma skin cancer: A univariable and multivariable Mendelian randomization study" was retracted in 2025. Reasons: unreliable results or conclusions; concerns about the methods; concerns about the peer review.

## ETHICS STATEMENT

This study did not involve any human participants or personal data. Therefore, ethics approval and consent to participate were not required.

## Supporting information

Supporting Information

Supporting Information

Supporting Information

Supporting Information

Supporting Information

Supporting Information

Supporting Information

## Data Availability

The data that support the findings of this study are available from the corresponding author upon reasonable request.

## References

[1] Meijs M , Herrera A , Acosta A , de Vries E . Burden of skin cancer in Colombia. Int J Dermatol. 2022;61: 1003‐1011.35141880 10.1111/ijd.16077

[2] Gosman LM , Țăpoi DA , Costache M . Cutaneous melanoma: a review of multifactorial pathogenesis, immunohistochemistry, and emerging biomarkers for early detection and management. Int J Mol Sci. 2023;24(21): 15881.37958863 10.3390/ijms242115881PMC10650804

[3] Arnold M , Singh D , Laversanne M , et al. Global burden of cutaneous melanoma in 2020 and projections to 2040. JAMA Dermatol. 2022;158:495‐503.35353115 10.1001/jamadermatol.2022.0160PMC8968696

[4] Sung H , Ferlay J , Siegel RL , et al. Global Cancer Statistics 2020: GLOBOCAN estimates of incidence and mortality worldwide for 36 cancers in 185 countries. CA Cancer J Clin. 2021;71:209‐249.33538338 10.3322/caac.21660

[5] Ding L , Gosh A , Lee DJ , et al. Prognostic biomarkers of cutaneous melanoma. Photodermatol Photoimmunol Photomed. 2022;38:418‐434.34981569 10.1111/phpp.12770

[6] Onesti CE , Josse C , Boulet D , et al. Blood eosinophilic relative count is prognostic for breast cancer and associated with the presence of tumor at diagnosis and at time of relapse. Oncoimmunology. 2020;9:1761176.32923121 10.1080/2162402X.2020.1761176PMC7458605

[7] Zhou X , Rong R , Xiong S , Song W , Ji D , Xia X . Integrated analysis to reveal potential therapeutic targets and prognostic biomarkers of skin cutaneous melanoma. Front Immunol. 2022;13:914108.36032150 10.3389/fimmu.2022.914108PMC9402985

[8] Kavitha P , Ayyappan G , Jayagopal P , et al. Detection for melanoma skin cancer through ACCF, BPPF, and CLF techniques with machine learning approach. BMC Bioinformatics. 2023;24:458.38053030 10.1186/s12859-023-05584-7PMC10699043

[9] Darcy CJ , Minigo G , Piera KA , et al. Neutrophils with myeloid derived suppressor function deplete arginine and constrain T cell function in septic shock patients. Crit Care. 2014;18:R163.25084831 10.1186/cc14003PMC4261583

[10] Benguigui M , Cooper TJ , Kalkar P , et al. Interferon‐stimulated neutrophils as a predictor of immunotherapy response. Cancer Cell. 2024;42:253‐265.e12.e212.38181798 10.1016/j.ccell.2023.12.005PMC10864002

The article "The causal relationships of granulocytes and melanoma skin cancer: A univariable and multivariable Mendelian randomization study" was retracted in 2025. Reasons: unreliable results or conclusions; concerns about the methods; concerns about the peer review.

[11] Carretero R , Sektioglu IM , Garbi N , Salgado OC , Beckhove P , Hämmerling GJ . Eosinophils orchestrate cancer rejection by normalizing tumor vessels and enhancing infiltration of CD8(+) T cells. Nat Immunol. 2015;16:609‐617.25915731 10.1038/ni.3159

[12] Moreira A , Leisgang W , Schuler G , Heinzerling L . Eosinophilic count as a biomarker for prognosis of melanoma patients and its importance in the response to immunotherapy. Immunotherapy. 2017;9:115‐121.28128709 10.2217/imt-2016-0138

[13] Pozorski V , Park Y , Mohamoud Y , et al. Neutrophil‐to‐eosinophil ratio as a biomarker for clinical outcomes in advanced stage melanoma patients treated with anti‐PD‐1 therapy. Pigment Cell Melanoma Res. 2023;36:501‐511.37903733 10.1111/pcmr.13109PMC11851330

[14] Davies NM , Holmes MV , Davey Smith G . Reading Mendelian randomisation studies: a guide, glossary, and checklist for clinicians. Bmj. 2018;362:k601.30002074 10.1136/bmj.k601PMC6041728

[15] Hemani G , Zheng J , Elsworth B , et al. The MR‐Base platform supports systematic causal inference across the human phenome. Elife. 72018.10.7554/eLife.34408PMC597643429846171

[16] Bowden J , Davey Smith G , Burgess S : Mendelian randomization with invalid instruments: effect estimation and bias detection through Egger regression. Int J Epidemiol. 2015;44: 512–525.26050253 10.1093/ije/dyv080PMC4469799

[17] Hartwig FP , Davey Smith G , Bowden J : Robust inference in summary data Mendelian randomization via the zero modal pleiotropy assumption. Int J Epidemiol. 2017;46:1985‐1998.29040600 10.1093/ije/dyx102PMC5837715

[18] Bowden J , Davey Smith G , Haycock PC , Burgess S . Consistent estimation in Mendelian randomization with some invalid instruments using a weighted median estimator. Genet Epidemiol. 2016;40:304‐314.27061298 10.1002/gepi.21965PMC4849733

[19] Burgess S , Scott RA , Timpson NJ , Davey Smith G , Thompson SG . Using published data in Mendelian randomization: a blueprint for efficient identification of causal risk factors. Eur J Epidemiol. 2015;30:543–552.25773750 10.1007/s10654-015-0011-zPMC4516908

[20] Cohen JT , Miner TJ , Vezeridis MP . Is the neutrophil‐to‐lymphocyte ratio a useful prognostic indicator in melanoma patients? Melanoma Manag 7: Mmt47, 2020.10.2217/mmt-2020-0006PMC747579732922729

[21] Cavallo F , Avallone G , Tartaglione C , Quaglino P , Ribero S . Attitudes, characteristics, and occupational‐related risk of skin cancer and cutaneous melanoma in the militaries: an observational, cross‐sectional, survey‐based study. Int J Dermatol. 2023;62:e167‐e168.36183247 10.1111/ijd.16439

[22] Wolchok JD , Chiarion‐Sileni V , Gonzalez R , et al. Long‐term outcomes with nivolumab plus ipilimumab or nivolumab alone versus ipilimumab in patients with advanced melanoma. J Clin Oncol. 2022;40:127–137.34818112 10.1200/JCO.21.02229PMC8718224

The article "The causal relationships of granulocytes and melanoma skin cancer: A univariable and multivariable Mendelian randomization study" was retracted in 2025. Reasons: unreliable results or conclusions; concerns about the methods; concerns about the peer review.

[23] Thrane K , Eriksson H , Maaskola J , Hansson J , Lundeberg J . Spatially resolved transcriptomics enables dissection of genetic heterogeneity in Stage III cutaneous malignant melanoma. Cancer Res. 2018;78:5970–5979.30154148 10.1158/0008-5472.CAN-18-0747

[24] Davey Smith G , Hemani G : Mendelian randomization: genetic anchors for causal inference in epidemiological studies. Hum Mol Genet. 2014;23:R89‐R98.25064373 10.1093/hmg/ddu328PMC4170722

[25] Emdin CA , Khera AV , Kathiresan S . Mendelian randomization. Jama. 2017;318: 1925–1926.29164242 10.1001/jama.2017.17219

[26] Xin Y , Yuan T , Wang J . The causal relationship between atopic dermatitis and brain cancer: a bidirectional Mendelian randomization study. Skin Res Technol. 2024;30: e13715.38646850 10.1111/srt.13715PMC11033834

[27] Xu W , Shen Y , Sun J , Wei D , Xie B , Song X . Causal role of immune cells in alopecia areata: a two‐sample Mendelian randomization study. Skin Res Technol. 2024;30: e13579.38221794 10.1111/srt.13579PMC10788640

[28] Shaul ME , Fridlender ZG . Neutrophils as active regulators of the immune system in the tumor microenvironment. J Leukoc Biol. 2017;102 343‐349.28264904 10.1189/jlb.5MR1216-508R

[29] Leliefeld PH , Wessels CM , Leenen LP , Koenderman L , Pillay J . The role of neutrophils in immune dysfunction during severe inflammation. Crit Care. 2016;20:73.27005275 10.1186/s13054-016-1250-4PMC4804478

[30] Sernicola A , Colpo A , Leahu AI , Alaibac M . Granulocyte apheresis: can it be associated with anti PD‐1 therapy for melanoma? Medicina (Kaunas). 2022;58(10):1398.36295558 10.3390/medicina58101398PMC9607554

[31] Karakonstantis S , Kalemaki D , Tzagkarakis E , Lydakis C . Pitfalls in studies of eosinopenia and neutrophil‐to‐lymphocyte count ratio. Infect Dis (Lond). 2018;50:163‐174.29070003 10.1080/23744235.2017.1388537

[32] Hirschhorn D , Budhu S , Kraehenbuehl L , et al. T cell immunotherapies engage neutrophils to eliminate tumor antigen escape variants. Cell. 2023;186:1432‐1447. e17.e1417, 2023.37001503 10.1016/j.cell.2023.03.007PMC10994488

[33] Matsumura Y , Kawarada Y , Matsuo M , et al. Retrospective analysis of neutrophil‐to‐lymphocyte ratio in patients with melanoma who received ipilimumab monotherapy or ipilimumab in combination with nivolumab in Japan. Biol Pharm Bull. 2023;46:427‐431.36858571 10.1248/bpb.b22-00750

[34] Ding Y , Zhang S , Qiao J . Prognostic value of neutrophil‐to‐lymphocyte ratio in melanoma: evidence from a PRISMA‐compliant meta‐analysis. Medicine (Baltimore). 2018;97:e11446.30045267 10.1097/MD.0000000000011446PMC6078713

The article "The causal relationships of granulocytes and melanoma skin cancer: A univariable and multivariable Mendelian randomization study" was retracted in 2025. Reasons: unreliable results or conclusions; concerns about the methods; concerns about the peer review.

[35] Wade RG , Robinson AV , Lo MCI , et al. Baseline neutrophil‐lymphocyte and platelet‐lymphocyte ratios as biomarkers of survival in cutaneous melanoma: a multicenter cohort study. Ann Surg Oncol. 2018; 25: 3341–3349.30066226 10.1245/s10434-018-6660-xPMC6132419

[36] Yang Z , Qi Y , Lai N , et al. Notch1 signaling in melanoma cells promoted tumor‐induced immunosuppression via upregulation of TGF‐β1. J Exp Clin Cancer Res. 2018;37:1.29301578 10.1186/s13046-017-0664-4PMC5755139

[37] Tasaki Y , Sugiyama Y , Hamamoto S , et al. Eosinophil may be a predictor of immune‐related adverse events induced by different immune checkpoint inhibitor types: a retrospective multidisciplinary study. Cancer Med. 2023;12:21666‐21679.37986680 10.1002/cam4.6724PMC10757154

[38] Proffer SL , Guo R , Demer AM , Peters MS . Eosinophils in metastatic melanoma. Hum Pathol. 2023;141:110–117.37574050 10.1016/j.humpath.2023.08.001

[39] Zahoor H , Barata PC , Jia X , et al. Patterns, predictors and subsequent outcomes of disease progression in metastatic renal cell carcinoma patients treated with nivolumab. J Immunother Cancer. 2018;6:107.30333065 10.1186/s40425-018-0425-8PMC6192175

[40] Ferrucci PF , Gandini S , Cocorocchio E , et al. Baseline relative eosinophil count as a predictive biomarker for ipilimumab treatment in advanced melanoma. Oncotarget. 2017;8:79809‐798155.29108362 10.18632/oncotarget.19748PMC5668095

